# Stem cell therapy for treating osteonecrosis of the femoral head: From clinical applications to related basic research

**DOI:** 10.1186/s13287-018-1018-7

**Published:** 2018-10-25

**Authors:** Rui Li, Qiu-Xia Lin, Xue-Zhen Liang, Guang-Bo Liu, He Tang, Yu Wang, Shi-Bi Lu, Jiang Peng

**Affiliations:** 1 Institute of Orthopedics, Beijing Key Laboratory of Regenerative Medicine in Orthopedics, Key Laboratory of Musculoskeletal Trauma & War Injuries, Chinese PLA General Hospital, Beijing, 100853 China; 2 The First Clinical Medical School, Shandong University of Traditional Chinese Medicine, Jinan, 250355 Shandong China

**Keywords:** Hip, Osteonecrosis, Cell therapy, Mesenchymal stem cells

## Abstract

Osteonecrosis of the femoral head (ONFH) is a refractory disease that is associated with collapse of the femoral head, with a risk of hip arthroplasty in younger populations. Thus, there has been an increased focus on early interventions for ONFH that aim to preserve the native articulation. Stem cell therapy is a promising treatment, and an increasing number of recent studies have focused on this topic. Many clinical studies have reported positive outcomes of stem cell therapy for the treatment of ONFH. To improve the therapeutic effects of this approach, many related basic research studies have also been performed. However, some issues must be further explored, such as the appropriate patient selection procedure, the optimal stem cell selection protocol, the ideal injection number, and the safety of stem cell therapy. The purpose of this review is to summarize the available clinical studies and basic research related to stem cell therapy for ONFH.

## Background

Osteonecrosis of the femoral head (ONFH) is a refractory disease that is characterized by compromised subchondral microcirculation, necrosis of the bone, and microfracture accumulation without sustained remodeling [1, 2]. ONFH is a global problem, and an estimated 20,000 to 30,000 new patients are diagnosed with osteonecrosis annually in the United States [3]; in addition, 8.12 million cases of nontraumatic ONFH are diagnosed annually among the Chinese general population aged 15 years and older [4].

Although total hip arthroplasty (THA) can provide satisfactory clinical outcomes for hip dysfunction patients, one challenge for surgeons is that ONFH occurs predominantly in patients aged 30 to 40 years. The outcomes of THA for these young and active patients are not ideal, primarily due to the limited lifetime and durability of the prosthesis. Thus, there has been an increasing focus on early interventions for ONFH that aim to preserve the native articulation. A wide variety of joint-preserving methods have been reported, including pharmacologic or physical treatment and surgical techniques ranging from core decompression (CD) to various vascularized and nonvascularized bone-grafting procedures [5]. However, the outcomes of these studies have varied. Thus, studies that aim to identify a better treatment are ongoing.

Stem cells are a group of cells with the ability to self-renew and form differentiated cells. These cells play important roles in development and disease. They are also important “seed” cells in the process of regenerative therapy. Stem cell research is currently focused mainly on adult stem cells, embryonic stem cells and induced pluripotent stem cells. Adult stem cells, which include mesenchymal stem cells (MSCs), have been reported as a promising approach for the regeneration of various tissues. MSCs were first described in human bone marrow and called bone marrow stem cells (BMSCs); these cells can be isolated from many other sources, including adipose tissue, the synovial membrane and the umbilical cord, in addition to the bone marrow [6, 7]. Since the injection of autologous MSCs combined with standard CD for treating ONFH was first described in 1993 and the first mid-term results were reported in 2002 [8], there has been an increased focus on this approach [9]; with the development of both the technology and the concept, stem cell therapy has been shown to be a promising approach for treating ONFH.

The aim of this paper is to present a review of current clinical and basic research related to stem cell therapy for treating ONFH.

## Outcomes in clinical applications

### General outcome

An increasing number of clinical studies have evaluated the therapeutic effect of stem cells on ONFH in recent years. Studies with high levels of evidence (Levels I and II) are shown in Table 1. Most of the authors demonstrated positive clinic outcomes, including reduced pain, improved function and motion, delayed progression or the avoidance of THA [10–17]. However, several researchers had reservations about this approach. Pepke et al. reported that there was no significant benefit from the additional injection of concentrated bone marrow aspirate compared with the effects of CD alone in the short term (Level of Evidence: I) [18]. In addition, several retrospective comparative studies (Level of Evidence: III) drew conclusions similar to those reported by Pepke [19, 20]. A recent meta-analysis showed that the implantation of autologous MSCs into the CD track, particularly in the early (precollapse) stages of ONFH, could improve the survivorship of femoral heads and reduce the need for hip arthroplasty [21]. Another meta-analysis (including eight randomized controlled trials) also demonstrated that compared with CD alone, the combination of CD with regenerative techniques provides a significant improvement in survivorship over time [9].

**Table 1:** Details of landmark study and clinical studies with high levels of evidence*

Type of study	Author	Journal	Publication Date	Technique	Sample Size	Age (years)	Staging	Etiology	Processing of MSCs	Number of Cells	Complications	Follow-up	Conclusions
Level IV (Landmark study)	Hernigou et al. [8]	Clin Orthop Relat Res	2002	CD + BMC implantation	A total of 116 patients (189 hips)	31 (16 to 61)	SteiInberg I: 59; SteiInberg II: 86; SteiInberg III: 12; SteiInberg IV: 32	Steroid: 31; Alcohol: 56; Idiopathic: 10; SCD: 64; Organ transplantation: 21; Others: 7	150-mL bone marrow aspirate to a concentrated myeloid sus- pension of approximately 30 mL of stem cells	The average total number of colony-forming units injected by hip was estimated to be 25 × 103 cells.	No specific complication.	7 years (5 to 11 years)	Higher risk of failure for patients with corticosteroid treatment and stage III-IV. Correlation between the greater number of progenitor cells and smaller lesions with better outcomes.
Level I	Pepke et al. [18]	Orthopedic Reviews	2016	Control group: CD alone Treatment group: CD + BMC implantation	Control group: 14 hips; Treatment group: 11 hips	Control group: 44.5 ± 3.3; Treatment group: 44.3 ± 3.4	ARCO II 25	Chemotherapy: 2; Immunosuppressive therapy: 4	12 ml of bone marrow concentrate suspension was concentrated from 200 to 220 mL of marrow havesed from the iliac crest.	118.9 × 106 cells/ml (a total of 10 ml was injected).	NR	24 months	No significant benefit from the additional injection of BMC in the short term.
Level I	Tabatabaee et al. [16]	J Arthroplasty	2015	Control group: CD alone Treatment group: CD + concentrated bone marrow aspirates	Control group: 14 hips; Treatment group: 14 hips	Control group: 26.8 ± 5.8; Treatment group: 31 ± 11.4	ARCO I 5; ARCO II 16; ARCO III 7	Steroid: 19; Idiopathic: 9	Bone marrow concentrate suspension concentrated from approximately 200 mL of bone marrow aspirate.	2 million cells/ml (injected volume was not reported).	No serious complications were noted in either of the clinical groups.	24 months	BMC injection with CD could be an effective therapy for the early stages of AVN; score improvement.
Level I	Mao et al. [15]	J Bone Mine Res	2015	Control group: Porous tantalum rod implantation; Treatment group: Porous tantalum rod implantation + intra-arterial injection of peripheral blood MSCs	Control group: 41 hips; Treatment group: 48 hips	Control group: 36.12 ± 11.34; Treatment group: 34.60 ± 11.50	ARCO I 18; ARCO II 52; ARCO III 19	Steroid: 31; Alcohol: 32; Idiopathic: 26	Injections of G-CSF for 4 days to mobilize PBSCs, and then, a collection process was performed.	Injected cells: 2.47 × 108 mononuclear cells, which contained 1.71 ± 0.7 × 106 CD34+ cells.	No complication was observed.	36 months	Combination treatment provides superior results regarding clinical outcomes such as pain, function, activity, and motion compared with biomechanical support alone.
Level I	Ma et al. [14]	Stem Cell Res Ther	2014	Control group: CD + autologous bone graft Treatment group: CD + autologous bone graft with BMC	Control group: 24 hips; Treatment group: 25 hips	Control group: 34.78 ± 11.48; Treatment group: 35.60 ± 8.05	Ficat I: 7; Ficat II: 32; Ficat III: 10	Steroid: 26; Alcohol: 7; Idiopathic: 12	Centrifuged and then loaded into the cylindrical bone.	The average number of bone marrow cells loaded into the cylindrical bone was approximately 3 × 109 nucleated cells.	No complication was observed.	24 months	Implantation of the autologous BMC graft combined with CD is effective to prevent further AVN. The stage of AVN might affect the outcome, while etiological factors do not.
Level I	Rastogi et al. [13]	Musculoskelet Surg	2013	Control group: CD and unprocessed bone marrow injection Treatment group: CD + isolated mononuclear cells	Control group: 30 hips; Treatment group: 30 hips	Control group: 33.0 ± 7.71; Treatment group:34.67 ± 7.02	NR	Steroid: 18; Alcohol: 8; Idiopathic: 26; Smoking: 8	Treatment group: 5 ml of isolated mononuclear cells (The entire procedure took 1 h). Control group: 30–50 ml of unprocessed bone marrow.	Treatment group: 1.1 × 108 cells. Control group: not reported.	No complications were noted in both group.	24 months	Control and treatment group scores show significant differences when compared with preoperative scores, without statistically significant inter-group differences in clinical scores.
Level I	Sen et al. [12]	J Arthroplasty	2012	Control group: CD alone Treatment group: CD + autologous bone marrow mononuclear cell	Control group: 25 hips; Treatment group: 26 hips	NR	ARCO I, II	Steroid: 14; Alcohol: 6; Idiopathic: 1; Pregnancy: 1; Cushing disease: 1; Trauma: 17	2 ml of mononuclear cells was havested from 120 to 180 ml of bone marrow aspirates in appromixmately 2 h.	Injected cells: 5 × 108 mononuclear cell to keep to keep the CD34 + cell count more than 5 × 107 .	No complications were observed.	24 months	BMC instillation can result in better clinical outcomes and hip survival, with only 1 THR in the treatment group vs 6 in the control group. Better outcomes in traumatic AVN than in non-traumatic AVN.
Level I	Zhao et al. [11]	Bone	2012	Control group: CD alone Treatment group: CD with cultured bone-marrow derived MSCs	Control group: 44 hips; Treatment group: 53 hips	Control group: 33.8 ± 7.7; Treatment group: 32.7 ± 10.5	ARCO IC 5; ARCO IIA 30; ARCO IIB 46; ARCO IIC 23	Steroid: 24; Alcohol: 19; Idiopathic: 30; Trauma: 20; Caisson disease: 11	10 mL of subtrochanteric bone marrow was aspirated and allowed to proliferate in vitro for two weeks.	Implanted cells: 2 × 106 cells.	No complications were observed.	60 months	Ex vivo expansion of bone marrow-derived MSCs and implantation provide significant improvements in pain and other joint symptoms and delay or avoid the progression of osteonecrosis and THA.
Level I	Gangji et al. [10]	Bone	2011	Control group: CD alone Treatment group: CD + BMC implantation	Control group: 11 hips; Treatment group: 13 hips	Control group: 45.7 ± 2.8; Treatment group: 42.2 ± 2.6	ARCO I 4; ARCO II 20	Steroid: 20; Alcohol: 2; Idiopathic: 2	Concentrated to a final volume of 49.7 ± 2.3 ml.	Contained 1.9 ± 0.2 × 109 mononuclear cells, including 1.0 ± 0.1% of CD34+ cells.	No complications were observed.	60 months	BMC implantation in the necrotic lesion provides better results in early osteronecrosis and delays its progression. Reduced pain and decreased volume of the necrotic lesion.
Level II	Houdek et al. [23]	Clin Orthop Relat Res	2018	A consecutive cohort, CD + BMC + PRP	A total of 22 patients (35 hips)	43 (22 to 66)	Pennsylvania Stage 1 or Stage 2	Steroid	60 to 120 cc of bone marrow was concentrated to 6 to12 cc of BMC	2.5 × 106 to 6.8 × 107 cells.	NR	3 years (2 to 4 years)	Successful results were seen when the nucleated cell count was high and the modified Kerboul grade was low.
Level II	Pilge et al. [49]	Ortho Rev.	2016	Control group: CD + iloprost iv. Treatment group: CD + iloprost iv. + BMC implantation	Control group: 10 hips; Treatment group: 10 hips	38.35 (15 to 58)	ARCO II: 12; ARCO III: 6; ARCO IV: 2	Steroid: 5; Chemotherapy: 6; Idiopathic: 8; Smoke: 1	60 ml of bone marrow aspirate was concentrated.	Between 7 and 10 mL.	No serious adverse reaction to iloprost infusion. Patients had flush symptoms and 2 patients complained of a mild headache during infusion.	30.6 (4–69) months	An improvement in clinical scores was shown in the treatment group but not in the control group.
Level II	Gangji et al. [17]	J Bone Joint Surg Am	2004	Control group: CD alone Treatment group: CD + BMC implantation	Control group: 8 hips; Treatment group: 10 hips	Control group: 48.8 ± 11.2; Treatment group: 40.9 ± 9.8	ARCO I: 2; ARCO II: 16	Steroid: 14; Alcohol: 2; Idiopathic: 2	Approximately 400 mL of marrow was obtained from the anterior iliac crest and concentrated to a mean final volume of 51 ± 1.8 mL.	2.0 ± 0.3× 109, including 1.0% ± 0.2% CD34+ cells.	No major side effects was observed. Two patients complained of pain at the site of the bone-marrow aspiration; coagulase- negative staphylococc was cultured form the bone marrow in one patient; A hematoma was observed at the site of the CD in another patient	24 months	CD + BMC provides significant decreases in the level of pain and other joint symptoms. The volume of necrotic lesions significantly improved only in the treatment group.

*High levels of evidence refers to Levels I and II; AVN, avascular necrosis of the femoral head; CD, core decompression; MSC, mesenchymal stem cell; BMC, bone marrow concentrate; ARCO, Association Research Circulation Osseous; SCD, sickle cell disease; G-CSF, granulocyte-colony stimulating factor; THA, total hip arthroplasty; NR, not reported

Thus, although some controversy exists, it seems that the general outcomes of the use of stem cells to treat ONFH are positive. The reasons for the different conclusions may be the heterogeneity among studies, including differences in patient selection, cell harvesting, cell processing, and cell delivery. Thus, these heterogeneities warrant further investigation.

### Patient selection

Numerous studies confirmed that the outcome of treatment was ascociated with patient condition. The most important factor may be the stage of ONFH. Ma et al. reported that the stage of ONFH might affect the outcome of stem cell therapy [14]. Hauzeur et al. reported that the implantation of bone marrow aspirate concentrate (BMAC) after CD did not produce any improvement in the evolution of stage III ONFH [22]. Thus, stage III and stage IV cases may be prone to poor outcomes, and early-stage (stage I or II) patients should be a more appropriate choice. In addition, Sen et al. [12] reported that patients with posttraumatic osteonecrotic hips had better outcomes than did patients with nontraumatic hips, which suggested that etiology is another a factor that affects clinical outcomes. Furthermore, Houdek et al. suggested that patients with a low modified Kerboul grade may achieve better results [23]. It seems that the stage, size, morphology and even etiology of ONFH may be important factors associated with the treatment outcome. Thus, to achieve better results, it is critical to select appropriate cases.

Moreover, it has been reported that aging is associated with decreases in the number of MSCs isolated from a donor and the proliferation ability of those cells [24, 25]. Stenderup et al. [26] found that although MSC function was decreased in cells isolated from older donors in vitro, this difference did not affect the ability of the cells to differentiate in vivo. The authors concluded that MSCs isolated from older donors maintained normal cellular function but showed a proliferative defect. In addition, Aksu et al. [27] found that sex may affect the differentiation potential of human adipose-derived stem cells. However, Sen et al. [12] reported that patient variables, such as sex differences, side of involvement, and opposite side involvement, had no effect on outcomes. Whether these factors influence the treatment efficiency in ONFH patients has not been well studied. Additional studies that are focused on subgroup analysis and the proper inclusion criteria for stem cell therapy in ONFH patients are needed in the future.

### Cell selection

Various types of MSCs have been used to treat ONFH, including bone marrow-derived MSCs (BMMSCs), adipose-derived MSCs (ADMSCs), allogeneic human umbilical cord-derived MSCs (hUCMSCs) and peripheral blood MSCs (PBMSCs). Among the various kinds of MSCs derived from different tissues, BMMSCs are the most commonly used type. BMMSCs are used mostly as bone marrow concentrate (BMC) and are more rarely cultured or used simply as bone marrow aspirates [9]. Rastogi et al. [13] compared isolated mononuclear cells with unprocessed bone marrow injections and found that there were considerable improvements in hip function, as measured by the Harris hip score, in both groups. There was a decrease in the lesion size in the processed isolated mononuclear cell group, and 3 of 30 hips in the unprocessed bone marrow injection group required total hip replacement. It seems that the more effective procedure had better outcomes than did unprocessed bone marrow injection for the treatment of ONFH.

In addition to BMMSCs, ADMSCs are another choice for cytotherapy in patients with ONFH. This method of acquiring MSCs is not only less expensive but also less invasive and painful than that used for bone marrow harvesting [28]. An in vitro study demonstrated that adipose-derived MSCs may provide a more robust growth rate and bone differentiation potential than bone marrow-derived MSCs [29]. As adipose-derived MSCs are more abundant and show a superior functional phenotype for this purpose, they may prove to be a more effective therapeutic approach. Although the results of these studies were promising, there is a lack of well-designed prospective in vivo clinical studies to further confirm this conclusion.

Moreover, it has been demonstrated that the osteogenesis and proliferation of MSCs are decreased in alcohol-induced and steroid-induced ONFH patients [30–33]. Therefore, the transfusion of autologous stem cells isolated from these patients may have different therapeutic effects. Thus, allogeneic stem cells derived from healthy humans may be an alternative for treating ONFH. Interestingly, there is evidence for the accumulation of low-immunogenicity MSCs, which allows the MSCs to be transplanted between human leukocyte antigen (HLA)-incompatible individuals [34]. hUCMSCs may be a good candidate for this approach, because umbilical cord (UC) collection is easy and ethically feasible. The yield of UCMSCs is high, and the cells have low immunogenicity. UCMSCs are easy to separate and can be amplified in vitro; placental UCMSCs can typically be passaged for 30–40 generations, while adult BMMSCs can grow only 6–10 generations with the same performance.

Cai et al. [35] evaluated the cotransplantation of autologous BMMSCs and allogeneic UCMSCs for treating ONFH and observed therapeutic effects without severe adverse effects at 12 months after transplantation. Chen et al. [36] analyzed the clinical effects of transplanting allogeneic hUCMSCs for the treatment of ONFH and achieved clear results with no obvious side-effects after a three-year follow-up. However, there were only 30 cases and 9 cases in the studies of Cai et al. and Chen et al., respectively. Studies with larger numbers of patients and longer follow-up times are needed to further evaluate the efficiency and safety of the use of allogeneic hUCMSCs in treating ONFH.

### Number of injected cells

The prevalence of connective tissue progenitors in the bone marrow in the iliac crests of patients was approximately one per 30,000 nucleated cells [37]. Hernigou et al. reported that according to the mean nucleated cell count per ml (18 × 10^6^ cells), the bone marrow harvested from the iliac crest by aspiration contained an average of approximately 600 progenitors per ml [38]. If expansion is performed in vitro, more cells will be harvested.

It was reported that good outcomes may be associated with high nucleated cell counts [20, 23]. However, the optimum number of cells for injection remains unknown. The average volume repair was 15 cm^3^ in a series of osteonecrosis patients, as indicated by MRI observations and histologic observations that demonstrated that the proportion of trabecular bone was 1/3 in the femoral head, with the other 2/3 being fat and hematologic cells [39]. Based on a mean bone matrix of 33% in cancellous bone, it was estimated that there are approximately 20 million osteoblasts or osteocytes per cm^3^ of new bone [39]. Thus, approximately 3 × 10^8^ (20 million cells/cm^3^ × 15 cm^3^) osteoblasts or osteocytes are needed for new bone repair. However, achieving an objective number of osteoblasts or osteocytes depends not only on the number of stem cells injected but also on how many times the stem cells can proliferate and how many cells can effectively differentiate into osteoblasts or osteocytes, especially in the ischemic and anoxic microenvironment of the necrotic area of the femoral head. On the other hand, whether the injection of more stem cells is better and whether there is a safe threshold for the maximum injection of stem cells remain unknown.

Based on current reported studies, except for patients injected with approximately 24 × 10^3^ to 25 × 10^3^ cells in early studies reported by Hernigou et al. [8, 40], the number of cell used in most other studies ranged from 10^6^ to 10^9^, and the most frequently used number was 10^8^ cells [11–13, 18, 20]. Thus, based on current data, the injection of 10^6^ to 10^9^ cells may be reasonable. However, the optimal number still needs to be investigated.

### Delivery techniques and combined treatment

Various techniques for cell delivery have been reported in recent studies, and such techniques were commonly combined with CD [10–12, 16, 18]. Other techniques included impaction allogeneic bone grafting [41, 42], autoiliac cancellous bone grafts [43, 44], porous tantalum rod implantation procedures [15], porous tantalum rod implantation combined with vascularized iliac grafting [45], interconnected porous calcium hydroxyapatite (IP-CHA) [46] and porous nanohydroxylapatite [47].

In addition to the topical application of MSCs in the necrotic zone of the femoral head, some studies also applied the MSCs through arterial injection. Cai et al. transplanted MSCs into the medial circumflex femoral artery, the lateral circumflex femoral artery or the obturator artery through digital subtraction angiography and observed a therapeutic effect on avascular necrosis of the femoral head (ANFH) without severe adverse effects [35]. Mao et al. reported the intra-arterial infusion of PBMSCs and found that this approach could enhance the efficacy of biomechanical support during the treatment of ONFH [15]. These two studies demonstrated that intra-artery infusion could be another effective way to treat ONFH. In addition, these studies also provided evidence that MSCs could effectively act on ischemic areas. However, determining whether the topical application or intra-arterial infusion of MSCs is more effective requires further investigation.

Some studies also combined local injection with platelet-rich plasma (PRP) [48], pharmacological treatments, such as intravenous iloprost [49] and oral bisphosphonates [19], or physical therapy, such as low-intensity pulsed ultrasound (LIPUS) [50]. Most of these studies reported satisfactory outcomes, but some studies had lower levels of evidence; thus, whether such combinations support better outcomes must be further confirmed. Moreover, comparisons between various methods have rarely been reported.

Note that, in general, regardless of which delivery technique and combined treatment were used, all of the approaches yielded improved results.

### Safety

One of the major concerns in cell therapy is safety. Stem cells have some features of cancer cells, including a long lifespan, relative apoptosis resistance, and the ability to replicate for extended periods of time. In addition, similar growth regulators and control mechanisms are involved in both cancer and stem cell maintenance. Therefore, stem cells may undergo malignant transformation, which is often seen as a key obstacle to the safe use of stem-cell-based medicinal products [51]. It was reported that the transplantation of embryonic stem cells may increase the risk of teratoma formation [52]. Other concerns, including immune rejection and genetic modification, also limit the clinical use of directly transplanted stem cells for ONFH.

After a review of current studies that used stem cells in the treatment of ONFH, we found that most studies reported that no severe complications were observed. Only a few studies reported that patients had complications, such as flushing, mild headache and fever [44, 49]. Thus, based on the current studies, it seems that the application of stem cells for the treatment of ONFH is relatively safe. However, additional studies and long-term follow-up are still needed to further confirm this conclusion.

In addition, for cell therapy, which requires cell expansion in vitro, the entire process must be supervised to ensure that the cells maintain their overall phenotype and functional potential and to ensure that the cultured cells remain untransformed with no microbiological contamination [51]. Thus, standardization with respect to the quantitative and qualitative characterization of cellular therapies may need to be established in the future.

## Advances in related basic research

### Rationale behind cell therapy

Although overall, clinical trials have achieved promising results, it is undeniable that a few studies were not valid. Thus, stem cell therapy remains controversial, which has limited its widespread use. Therefore, to improve the treatment effect of stem cell therapy, many exploratory studies, including cell experiments and animal experiments, have been performed.

A major concern of stem cell therapy is the fate and potential osteogenic activity of MSCs in the ischemic and hypoxic microenvironment at the osteonecrotic site, where the apoptosis of bone cells may occur [53]. It was reported that transplanted stem cells exhibit a low survival rate in ischemic tissue [54].

Yan et al. [55] transplanted autologous MSCs after decompression in traumatic dog models. They found that green fluorescent protein (GFP)-labeled MSCs were present in the necrotic area up to 12 weeks after transplantation, and their number increased from 15% in the 2nd week to 38% in the 12th week. Immunohistochemical staining for osteocalcin was positive in 90% of the GFP-labeled MSCs in vivo. The percentages of trabecular bone volume were 9.36% and 8.42% in the 2nd week (*p* > 0.05), 22.82% and 14.72% in the 8th week, and 31.08% and 20.66% in the 12th week for the MSC-treated and control groups, respectively, and new trabecular bone in the MSC-transplanted group was significantly increased compared to that of the saline (control) group in the 8th and 12th weeks. This finding demonstrated that the transplanted MSCs could survive, proliferate, and differentiate into osteoblasts directly.

Jin et al. [56] drew a conclusion similar to that reported by Yan. They found that intra-arterially infused MSCs could migrate into the necrotic field in the femoral head and differentiate into osteoblasts, improving necrosis of the femoral head.

Moreover, Ciapetti et al. demonstrated that proliferation, colony formation and osteogenic commitment are not hampered by a low-O_2_ microenvironment [57]. In their study, the cells were expanded and induced to undergo osteogenic differentiation under a 2% pO_2_ atmosphere (hypoxia), in contrast to their behavior under the standard 21% pO_2_ atmosphere (normoxia). Those authors found that both proliferation and colony-forming ability were significantly enhanced in hypoxia-exposed BMMSCs compared with those of BMMSCs grown under normoxic conditions. The expression of bone-related genes, including alkaline phosphatase, type I collagen, and osteocalcin, was significantly increased under hypoxic conditions. Moreover, mineral deposition after osteogenic induction was not hampered and was even enhanced in some cases under low oxygen tension. These findings suggest that MSCs can survive and maintain their function in a hypoxic microenvironment.

Fan et al. [58] found that compared with BMMSCs from normal rabbits, BMMSCs from osteonecrotic rabbits showed a significantly reduced proliferative ability, reduced expression of stemness genes, decreased osteoblast formation, and increased adipocyte formation. However, after low-oxygen (2%) treatment, BMMSCs from osteonecrotic rabbits showed not only increased proliferation and osteogenic potential but also decreased adipogenic potential. Further, those authors demonstrated that the transplantation of 2% O_2_ versus 20% O_2_ MSCs after CD resulted in an increase in angiogenic function and a decrease in local tissue apoptosis in a rabbit model. Hypoxia-preconditioned BMMSCs could reverse the impairment of osteonecrotic BMMSCs and enhance their therapeutic effects [59]. Other studies drew the similar conclusion that an osteogenic phenotype can be promoted if MSCs are exposed to hypoxia during the initial steps of differentiation [60–62].

Thus, transplanted cells can survive, proliferate, and differentiate into osteoblasts in osteonecrotic areas in animal models. Interestingly, a low-O_2_ microenvironment does not seem to harm MSCs and even promoted the osteogenic phenotype in cellular experiments; these findings must be confirmed in humans.

### Subpopulations of MSCs

A definition for MSCs was provided by the International Society for Cellular Therapy in 2006 [63]. First, MSCs must be plastic adherent when maintained under standard culture conditions. Second, MSCs must express CD105, CD73 and CD90 and lack the expression of the CD45, CD34, CD14 or CD11b, CD79alpha or CD19 and HLA-DR surface molecules. Third, MSCs must differentiate into osteoblasts, adipocytes and chondroblasts in vitro. Although this definition is currently widely accepted, evidence that MSC subpopulations may feature distinct characteristics and regeneration potentials has been reported, and different subpopulations have distinct potentials to promote differentiation into osteoblasts or chondrocytes [64].

Levi et al. [65] demonstrated that compared with either CD105(high) or unsorted cells, FACS-sorted CD105(low) ADMSCs were significantly enhanced in osteogenic differentiation and bone regeneration; this effect is likely due to reduced TGF-beta1/Smad2 signaling. Additionally, Leyva-Leyva et al. [66] observed that CD105- cells showed stronger expression of secreted protein acidic and rich in cysteine (SPARC) and osteonectin, which was associated with more effective calcium deposition, than did CD105+ cells. Furthermore, through in vivo trials, it was demonstrated that grafts containing CD105- cells promoted adequate graft integration, improved host vascular infiltration, and facilitated efficient repair through intramembranous ossification. By contrast, grafts containing CD105+ cells showed abundant fibrocartilaginous tissue and deficient endochondral ossification [67].

While conflicting data have been reported for BMSCs, Aslan et al. [68] found that in the bone marrow, CD105+ cells displayed significantly more fibroblast colony-forming units than did unseparated mononuclear cells. Similarly, Jarocha et al. [69] reported that expanded CD105 and CD271 populations possess higher expression levels of RUNX2 and OCN.

CD90 is another marker for subpopulation selection. Yamamoto [70] found that CD90+ cells are more capable of forming bone both in vitro and in vivo. In addition, CD90 may be a more effective marker than CD105 for isolating a highly osteogenic subpopulation. Rada et al. [71] reported that the cells isolated with an anti-CD90 antibody (ab), an anti-CD49d ab and an anti-p75 ab exhibited a high osteogenic differentiation potential but demonstrated the lowest chondrogenic differentiation potential. On the other hand, the cells isolated with an anti-CD73 ab exhibited a high chondrogenic differentiation potential but the lowest osteogenic potential.

In addition, Harumichi et al. [72] reported that although significant differences in proliferation capacity were not seen, the adipogenic and osteogenic differentiation capacities were higher in aldehyde dehydrogenase (ALDH)-high subpopulations than in ALDH-low subpopulations. All these studies revealed that osteogenic potential is related to different subpopulations.

To date, preclinical and clinical studies of ONFH treatments used unsorted MSCs, which may consist of various cell subpopulations; this factor may be one of the most important reasons for the inconsistent results of previous studies. Thus, the accurate selection of a subpopulation may enhance treatment efficiency for ONFH and may be a direction for future research.

### Gene-modified MSCs

Some studies have also focused on the use of genetic engineering to modify MSCs, such as bone morphogenetic protein-2 (BMP-2), basic fibroblast growth factor (bFGF), hepatocyte growth factor (HGF), vascular endothelial growth factor (VEGF), calcitonin gene-related peptide (CGRP) or their combinations.

Tang et al. [73] used BMP-2-modified BMMSCs to repair experimentally induced ONFH in goats and obtained good results. Pend et al. demonstrated that BMP-2- and bFGF-modified BMSCs could successfully repair ONFH in a dog model by promoting bone formation and angiogenesis [74]. VEGF alone or combined with BMP-2-modified MSCs also yielded positive results in dog and rabbit experiments [75, 76].

In addition, the ability of HGF, a pleiotropic cytokine, to exert potent mitogenic effects and promote nutrient absorption and utilization to facilitate tissue repair in the liver, heart and muscle was also evaluated. Wen et al. [77] demonstrated that the combination of CD and the transplantation of HGF-transgenic autologous BMSCs enhanced blood vessel regeneration and bone reconstruction in a rabbit ANFH model. This positive outcome was also confirmed by Pan et al. [78].

Gene-modified MSCs may be a promising technique for improving treatment efficiency in ONFH patients. However, all these results were obtained in animal experiments. The efficiency and safety of these approaches in ONFH patients require further evaluation.

### MSC-derived exosomes for cell-free therapy

It was originally thought that MSCs exert their therapeutic effect by migrating to sites of damage, engrafting, and subsequently differentiating into the desired cells for tissue regeneration. However, accumulated evidence has indicated that the therapeutic benefit of MSCs is attributable not only to their differentiation but also to the factors they secrete [79–81]. In addition to growth factors, cytokines, chemokines, and bioactive lipids secreted by stem cell therapeutics, cells can communicate with neighboring cells or with distant cells through the secretion of extracellular vesicles (EVs). EVs are composed of a lipid bilayer that contains transmembrane proteins and encloses cytosolic proteins and RNA. Cells can secrete different types of EVs, such as exosomes and microvesicles (MV), which have been classified according to their subcellular origins [82]. Exosomes are vesicles that are smaller than 150 nm in diameter and enriched in endosome-derived components [83].

Guo et al. demonstrated that exosomes from human synovial-derived MSCs could prevent glucocorticoid-induced ONFH in rats by enhancing proliferation and antiapoptotic effects [84]. Liu et al. further reported that exosomes secreted from human-induced pluripotent stem cell-derived MSCs could prevent ONFH by promoting angiogenesis [85].

This cell-free treatment plays an increasingly important role in regenerative therapy. However, unlike pharmaceutical treatments that deliver a single agent at a specific dose, MSCs are site-regulated and secrete bioactive factors and signals at variable concentrations in response to local microenvironmental cues [86]. Thus, whether MSC-derived vesicles can fully replace MSCs must be further evaluated.

In addition, the potential risks of using exosomes should be considered. Accumulating evidence has indicated that cells communicate via the release and delivery of microRNAs (miRNAs) packed into tumor-released (TR) exosomes [87]. It was also reported that exosome vehicles could transfer toxic proteins associated with neurodegenerative diseases [88]. Thus, the safety of using MSC-derived vesicles must also be evaluated.

Finally, there is much work to be done before MSC-derived vesicle therapy can be used clinically, including standardized production, vesicle characterization, improved isolation and yield optimization, reproducibility, the development of an assay for potency, and a determination of the doses for particular clinical indications.

## Conclusion

Extensive research activities over the last decade have explored the potential of MSCs and have shown promising results in both animal experiments and clinical applications. Although some controversy exists, it seems that the general outcomes of the use of stem cells to treat ONFH are positive in terms of not only efficiency, but also safety.

For clinical applications, the different conclusions may be due to the heterogeneity among studies. It seems that patients in ARCO I and ARCO II stages and patients with a low modified Kerboul grade are good candidates for this technique. BMMSCs were still the most commonly used cells, while other types of stem cells, such as ADMSCs, show a more promising prospect, with a robust growth rate and bone differentiation potential, and could be considered as an alternative to BMMSCs. In addition, it was reported that the good outcomes may be associated with high nucleated cell counts. Although the most proper number of cells for injection was not determined, based on the current available data, injection of 10^6^ to 10^9^ cells may be reasonable. Further clinical applications should be aware of the appropriate patient selection procedure, the optimal stem cell selection protocol and the ideal injection number to achieve better outcomes.

For the related basic research, inspiring advanced progress has been made. Preconditioning of MSCs and accurate selection of a subpopulation may enhance treatment efficiency for ONFH. Use of genetic engineering to modify MSCs, such as BMP-2 and VEGF, also constituted good attempts to use MSCs more efficiently. Recently, cell-free treatment has played an increasingly important role in regenerative therapy and may develop as an alternative to stem cell therapy. However, much work must be done before these experimental approaches can be applied in clinical practice, in terms of not only efficiency, but also safety. Standardization with respect to the quantitative and qualitative characterization of cellular therapies is urgently needed in the future.
